# Development of Nanoemulsions for Wound Dressings Containing *Cassia alata L*. Leaf Extraction

**DOI:** 10.1155/2022/4282678

**Published:** 2022-10-11

**Authors:** Surat Sangkaew, Smith Wanmasae, Kingkan Bunluepeuch, Tassanee Ongtanasup, Siriwan Srisang, Chawan Manaspon, Philaslak Pooprommin, Komgrit Eawsakul

**Affiliations:** ^1^School of Medicine, Walailak University, Nakhon Si Thammarat 80160, Thailand; ^2^School of Allied Health Sciences, Walailak University, Thasala District, Nakhon Si Thammarat 80160, Thailand; ^3^Energy Engineering Division, Department of Engineering, King Mongkut's Institute of Technology Ladkrabang, Prince of Chumphon Campus, Chumphon 86160, Thailand; ^4^Biomedical Engineering Institute, Chiang Mai University, Chiang Mai 50200, Thailand; ^5^School of Allied Health Sciences and Research Excellence Center for Innovation and Health Products (RECIHP), Walailak University, Nakhon Si Thammarat 80160, Thailand

## Abstract

Natural polymer-based hydrogel films possess considerable potential for use in biomedical applications and are excellent for wound healing. The purpose of this research was to use ionic crosslinking to improve the mechanical characteristics, absorption of fluid in the wound, and drug release behavior of *Cassia alata L*. (CA) extract loaded niosomes (CANs) that were incorporated in an alginate-pectin film (A/P). Then, chemically crosslinked A/P hydrogels were obtained by immersing them in different concentrations of calcium chloride (CaCl_2_) (0.5–1% w/v) for 15–120 s. The degree of crosslinking was controlled by both contact time and CaCl_2_ concentration. The optimal crosslinking conditions were 1% CaCl_2_ for 15 seconds. In this study, the following features of the hydrogel films were investigated: physical properties, morphological characteristics, drug loading, *in vitro* drug release, antibacterial activity, wound healing activity, cytocompatibility profiles, and hemocompatibility. The crosslinked hydrogel films maintained their physical integrity during use, with the 1% film attaining the best results in the shortest period (15 sec). Then, *in vitro* drug release from the films was examined. Crosslinking was observed to prolong the release of the CA extract from the hydrogel film. Finally, a cell viability experiment was conducted to evaluate the cytotoxicity profile. The A/P composite film exhibited excellent wound dressing qualities and good mechanical properties in preformulation testing. The *in vitro* drug release profile indicated that the A/P created a regulated drug release profile, and the cell viability experiment revealed that the film was nontoxic and hemocompatible. A/P composite films can be produced using CAN extract as a possible wound dressing. However, further studies in animals and humans are required to determine both safety and effectiveness.

## 1. Introduction

The skin is the body's largest and most burdened organ. It covers an area of over 7,600 sq cm (3000 sq inches) in ordinary individuals and accounts for 15% of their estimated body weight [1]. The skin is a dynamic tissue. It performs a variety of critical activities that not only defend the body from external harm and pathogens but also help to maintain the body's balance [2]. Cells and biological substances heal wounds. Processes include inflammation [3], cell proliferation, and tissue remodeling. Wound healing begins with cell division and proceeds to protrusion and migration before culminating in wound enclosure [4]. The goals of wound healing treatment are to repair wounds in the shortest period possible with the minimum level of pain and to rebuild the tissue [5–7]. In Thailand, wound healing using plant materials is commonly employed to treat gastric ulcers, burns, and skin problems [8]. Several Thai herbal plants have been discovered to have wound-healing properties and are being developed as a wound-healing alternative [9]. A wound infection hinders healing, causes abnormalities in the wounded tissue, and may even lead to death [10]. Infections require powerful antibiotics. Antibiotic-resistant microorganisms often impose a financial burden on patients. A technology that successfully restricts microbial growth, reduces antibiotic resistance, and is safe for humans is needed [11].

The search for herbal cures or plants has become increasingly important as the number of natural therapies increases [12]. Natural components have a role in medicine development [13]. Studies assessing the bioactivity of herbal medicines provide evidence for traditional applications and medication development. Medicinal plants are significant in economically deprived areas for treating sickness [14]. Thailand and Southeast Asia have historically employed medicinal herbs as alternative medicines [15, 16].

Plants, plant fibers, and animal fats were initially used to prepare wound dressings [17]. Existing approaches allow synthetic and natural materials to be utilized for multifunctional wound dressings [18]. Alginate is a hydrophilic, natural polyanionic polymer derived from brown marine algae that is considered a less expensive, nontoxic, and biocompatible biomaterial [19]. Alginate has a long history of usage in medicine, including tissue engineering, dental implant materials, and wound dressing [20]. However, because of its poor mechanical qualities, alginate is mixed with pectin to improve its mechanical properties [21]. Pectin is a hydrophilic and polyanionic polymer derived from fruit and vegetable pomace byproducts. Pectin is widely used as a wound dressing [22]. Alginate [23] and pectin-based hybrid hydrogels are appealing for wound dressing applications [24].

Although these polymers are nontoxic and biocompatible [25, 26], their antibacterial activities for avoiding wound infection are inadequate [27, 28]. Thus, an antibiotic wound dressing is needed. In fact, according to the study by Meenupriya et al. [29], *Cassia alata L*. (CA) has been used to treat skin infections and for wound healing for millennia. However, because bacterial inhibition lasts only a short time, the development of antibacterial agents for long-term bacterial inhibition is critical. The use of polymers as a drug carrier promotes the prolonged and regulated release of antibiotics, which might help to prevent long-term infections [30].

Niosomes are one of the most promising drug delivery carriers in numerous subcategories due to their qualities, such as excellent drug encapsulation and nontoxicity [31]. Niosomes are vesicular nonionic surfactant systems in which chemicals are loaded into vesicles. Nonionic surfactants such as Span or Tween, as well as cholesterol, are used to generate vesicles with a sonication process [32, 33]. Niosomes have been utilized for a variety of purposes, including targeted, long-term, and controlled substance release [34].

CA which has the common Thai name of “Chum Hed Thes,” belongs to the Leguminosae family and has been used to treat skin diseases; as an antihelminthic, antibacterial, laxative, and diuretic agent; to treat abscesses and wounds; for healing; and as a treatment for uterine disorders [35]. Therefore, CA is an interesting plant for use in antimicrobial and wound healing assays. The integration of this plant extract into niosomes improves the physical characteristics, antibacterial capabilities, and wound healing properties, making it a good alternative for wound healing. In a study of the active compounds of CA, the main active anthraquinones were rhein, aloe-emodin, emodin, chrysophanol, and physcion [36], and the main flavonoid was kaempferol. These substances inhibit the growth of bacteria [37] and inflammation [38].

The aim of the study was to develop herbs that would produce value and maximize their use by administering niosomes as a control for the release of active compounds of CA, which are effective at inhibiting bacterial growth for a long time period and do not affect fibroblast cells and red blood cells. Therefore, this study is the first to use a wound dressing prepared from sodium alginate and pectin (A/P) incorporating the CA extract in the niosome for controlled drug release.

## 2. Materials and Methods

### 2.1. Materials

Chloroform was obtained from Thai Oil Co. Ltd. (Thailand). Sodium alginate and pectin were purchased from Sigma-Aldrich Company. Dimethyl sulfoxide (DMSO) was purchased from Sigma-Aldrich (Germany). Mueller Hinton Agar (MHA) and trypticase soy agar (TSA) were obtained from Difco, Bacto Dickinson, Spark (USA). Oxacillin paper discs were purchased from Oxoid Limited (UK). Oxacillin sodium salt was purchased from Fluka, Sigma-Aldrich (Denmark). Dulbecco's modified Eagle's medium (DMEM), fetal bovine serum (FBS), 0.25% trypsin EDTA, trypan blue, phosphate-buffered saline (PBS), penicillin, streptomycin, 3-(4,5-dimethylthiazol-2-yl)-2,5-diphenyltetrazolium bromide (MTT), glycerin, Span 60, and cholesterol were purchased from Gibco® (Life Technologies, Paisley, Scotland). RCI Labscan Ltd. (Bangkok, Thailand) provided all of the solvents.

### 2.2. Plant Collection, Authentication, and Extraction

CA leaves were collected from Walailak University, Thasala district, Nakhon Si Thammarat Province, Thailand. The collected medicinal plant samples were identified by Komgrit Eawsakul, a Thai traditional medicine doctor, based on the plant identification handbook of the Royal Botanic Garden. Samples were deposited at the Department of Applied Thai Traditional Medicine, School of Medicine, Walailak University, Thailand. The collected fresh leaves were washed and dried at 55°C for 24 hours in the oven and mashed with a grinder. Then, the sample was boiled with water at 80°C. Finally, the extract was filtered and evaporated with a freeze dryer. The crude extract was stored at 4°C until the determination of bioactivities.

### 2.3. Calibration of CA Concentrations

A solution of CA extract (45 mg/ml) prepared in deionized water (DI) was subjected to spectrometry using a UV spectrometer by scanning wavelengths ranging from 200 to 600 nm. *λ*_max_ of ME was determined. The *λ*_max_ values of CA, which are 286 and 288 nm, were observed at pH 7.4 and 5.5, respectively, as shown in Figure 1. The freeze-dried powder of CA was dissolved DI at various concentrations (0, 50, 100, 200, 300, 400, and 500 *µ*g/ml). The standard curve of the CA solution was generated by detecting the absorbance at 286 and 288 nm with a spectrophotometer.

### 2.4. Preparation of CA Extract-Loaded Niosomes (CANs)

The thin-film hydration method was used to prepare niosomes with Span 60 **(**nonionic surfactant**)** and cholesterol. First, different proportions of Span 60 and cholesterol **(**1**:**1, 2**:**1, 3**:**1, and 4**:**1) were dissolved in chloroform (Table 1). The mixture was then agitated for 15 minutes before the chloroform was evaporated, creating a thin layer coating on a glass vial. The thin film layer was immersed in the CA solution **(**1 mg/ml**)** and agitated for 30 minutes, while the blank niosomes were hydrated in DI water. Afterward, probe sonication was performed for 30 seconds at 80% amplitude to construct the niosomes, which were stored at 4°C.

### 2.5. Physical Characterization of CAN

#### 2.5.1. Analysis of the Size and Polydispersity Index (PDI)

After niosome preparation, the niosome size, PDI, and zeta potential were determined by performing dynamic light scattering (Zetasizer Nano ZS, Malvern, UK) at 25 ± 0.1°C. The inverse Laplace transformation approach was used to extract the mean size and standard deviation (S.D.) from the instrument fitting data [39, 40]. The PDI indicates the quality of the dispersion size, with values smaller than 0.3 indicating good measurements and high-quality colloids. Each experiment was performed in triplicate.

#### 2.5.2. Determination of the Vesicle Charge

Following niosome production, samples (20 *µ*l) were diluted with 2 ml of DI water and filtered using Whatman No. 42 ashless filter paper. The zeta potential of each sample was measured six times, and the results were computed automatically using the Smoluchowski equation with a Zetasizer (Malvern Zetasizer Nano ZS, Malvern Instruments, UK) analyzer [33, 41, 42].

#### 2.5.3. Characterization of Drug Loading

The amount CA loaded in niosomes was determined by centrifugation. The white precipitate of the niosomes was removed by centrifugation at 5,000 rpm for 15 min at 4°C [43]. Then, the supernatant was filtered through a centrifuge filter (MWCO = 50 kDa) to eliminate the free drug. The samples were dried using a freeze-dryer. The drug loading content, encapsulation efficiency (EE), and yield of the dried samples were determined using the following equations:

(1) $$\begin{array}{c} \text{\% drug loading content}=\frac{\text{amount of drug in niosomes}}{\text{theoretical amount of nanoparticles }}\times 100, \end{array}$$

(2) $$\begin{array}{c} \text{\% drug loading efficiency}=\frac{\text{amount of drug in niosomes}}{\text{initial amount of drug in the system}}\times 100, \end{array}$$

(3) $$\begin{array}{c} \text{\% yield}=\frac{\text{practical total amount of nanoparticles}}{\text{theoretical total amount of nanoparticles}}\times 100. \end{array}$$

#### 2.5.4. *In Vitro* Evaluation of CA Release from Niosomes

Niosomes carrying drugs were placed in a dialysis bag (MWCO, Spectrum Labs, USA) with a molecular weight cutoff of 15 kDa. The bag was submerged in phosphate-buffered saline (PBS, pH 5.5, and 7.4) and incubated at 37°C and 90 rpm in an incubating shaker. At regular intervals, 15 ml of buffer solution (PBS) was replaced with 15 ml of fresh PBS. Free CA levels were also measured. The amount of drug released in the collected liquid was measured using UV-vis spectroscopy.

### 2.6. Preparation of a CAN-Incorporated Alginate and Pectin (A/P) Hydrogel

#### 2.6.1. Synthesis of A/P Hydrogels

The solvent-casting process was used to prepare alginate and pectin (A/P) films. The 1**:**1 ratio of sodium alginate (SA) to pectin (P) was achieved by dissolving the particles in DI water with mechanical agitation at 900 rpm until they were completely dissolved. During the manufacturing of the SA-P solution, the plasticizer agent glycerol was added at a rate of 15% (w/w), depending on the weight of the SA-P powder. After ultrasonication for 15 min, the solutions were degassed for 12 hours. Ten milliliters of the solution were cast into Petri dishes (diameter = 10 cm) to create SA-P films with glycerol. The films were then dried for two days at 55°C under controlled humidity (50%) conditions until completely dry. Dry film samples with appropriate dimensions were cut and immersed in 6 ml of 0.5% and 1% **(**w/v**)** CaCl_2_ aqueous solutions for 15, 30, 60, and 120 s to generate thin hydrogels with a good appearance and strength, as shown in Figure 2. Before use, the hydrogels were rinsed with distilled water and dried at 55°C until they reached a consistent weight.

#### 2.6.2. Preparation of CAN-Incorporated A/P Hydrogels

Since the niosomes containing a 1:1 ratio of Span 60 and cholesterol possessed a good percentage of drug loading and percent yield, as well as a high EE among the nanoemulsions, the 1:1 ratio was subsequently selected for further wound dressing formulation. Wound dressings were prepared using Span 60, cholesterol, SA, P, glycerin, crude extract, and purified water. When preparing the wound dressing formulation, glycerin was chosen to dissolve the crude extract. Glycerin is nontoxic, has good biocompatibility, and is widely used in the food, cosmetics, and pharmaceutical industries. A suitable volume of the CA solution was gradually added to the alginate solution until the final A/P/CA proportions (v/v) were 85:15 to generate the A/P/CA films. Afterward, the mixture was agitated for 30 minutes at 600 rpm, and 10 ml were poured onto Petri dishes. The films were dried for two days at 55°C under controlled humidity (50%) until they were completely dry. Dry film samples of appropriate diameters were cut and submerged in a 6 ml of an aqueous solution composed of 1% (w/v) CaCl_2_ for 15 seconds. The hydrogels were cleaned with distilled water and dried at 55°C until they attained a constant weight before being utilized.

#### 2.6.3. Analysis of the Swelling Percentage

The swelling behavior of the A/P film was studied in phosphate-buffered saline (PBS 7.4). Each film was immersed in 5 ml of PBS. The swelling experiments were conducted at room temperature by placing the samples in PBS. PBS was separated in each sample. At the scheduled time points, the samples were retrieved and quickly blotted twice on a Kimwipe tissue. The specimens were immediately weighed on an analytical balance that is accurate to 10^−4^ g. The blotting and weighing process was performed within 1 min for each sample. The initial wet weight was designated Wo, and the wet weight (W) during the immersion experiment was recorded at designated time points. The swelling ratio was calculated using equation (4). Samples were tested in groups of three. Averages and standard deviations are reported.

(4) $$\begin{array}{c} \text{\% swelling}=\frac{W}{W_{o}}\times 100. \end{array}$$

### 2.7. Biological Properties of CA Leaf Extracts

#### 2.7.1. Antimicrobial Activities

*(1) Agar Disc Diffusion Method*. The agar disc diffusion method was used to screen the antimicrobial activity (22). The crude extract was dissolved in distilled water and then diluted to a concentration of 200 mg/ml **(**2 mg/disc). The positive controls were 1 *µ*g/disc of oxacillin for *Staphylococcus aureus* (ATCC 25923) and *Staphylococcus epidermidis* (TISTR 517). Distilled water was used as a negative control.

*(2) Broth Microdilution Method*. The broth microdilution method was used to determine the antimicrobial activity (23). The crude extract was dissolved and diluted with distilled water at concentrations ranging from 0.25 to 16 mg/ml. The positive control oxacillin was prepared similarly to the samples and used for *S. aureu*s (ATCC 25923) and *S. epidermidis* (TISTR 517). Distilled water was used as a negative control. The experiment was performed in a 96-well plate, and two-fold dilutions were prepared directly in wells. Fifty microliters of the sample solution (dilutions ranging from 0.25 to 16 mg/ml) was added to wells 1 to 8 of the dilution series. The final concentration of the inoculum in each well was 5 × 10^5^ CFUs/ml.

#### 2.7.2. Cytotoxic Activity

The cytotoxic activity toward normal cells was determined using the sulforhodamine B (SRB) colorimetric assay [44]. Normal cells were obtained from the mouse fibroblast cell line (L929) passage No. 6. The sample was dissolved in distilled water at different concentrations (0.75–100 *µ*g/ml). Next, 5 × 10^3^ cells were added to each well and incubated for 24 hours. Then, the media were removed, replaced with fresh media, and incubated for 72 hours. Afterward, the cells were fixed with 10% trichloroacetic acid (TCA) and incubated for 1 hour at 4°C. Then, 100 *μ*l of 10 mM Tris base (pH 10.5) was added to each well and shaken to dissolve the SRB crystals until complete dissolution. Cell growth was determined by measuring the absorbance at 492 nm. Distilled water was used as a negative control in this study. The percent cytotoxicity was calculated using the following equations:

(5) $$\begin{array}{c} \text{\% of cell growth}=\left[\frac{\left({\text{OD}}_{492}\text{ of control}-{\text{OD}}_{492}\text{ of sample}\right)}{{\text{OD}}_{492}\text{ of control}}\right]\times 100\text{,} \end{array}$$

(6) $$\begin{array}{c} \text{\% cytotoxicity}=100-\text{ \% of cell growth.} \end{array}$$

#### 2.7.3. Cell Proliferation Assay

HDF cell proliferation tests were conducted in 96-well plates (1 × 10^4^ cells/well), and DMEM was used for cell culture. The cells were treated with different concentrations of the CA extract (0.75–100 *µ*g/ml) in 100 *µ*l of DMEM for 24 hours at 37°C in a humidified 5% CO_2_ atmosphere. Nontreated cells were used as a control. The cells were washed with PBS after 24 hours and then 100 *µ*l of fresh medium were added. Cell proliferation was evaluated using the MTT assay (10 *µ*l, 5 mg/ml) [45].

#### 2.7.4. Cell Migration (*In Vitro* Scratch Wound Healing Assay)

HDFs were seeded in 24-well plates (5 × 10^4^ cells/well) and incubated with at 37°C and 5% CO_2_ for 24 hours before analyzing cell migration. Afterward, a wound was created in the monolayer of cells using a 1,000 *µ*l sterile pipette tip. Then, the cell culture media were removed and cells were washed with PBS. When fresh medium was added, wound dressings were applied at various concentrations (1.56–6.25 *µ*g/ml). Photographs were captured on day 0, day 1, day 2, and day 3 and analyzed using ImageJ computing software (Nikon Co. Ltd., Japan). Three randomly determined points by the side of the wound margin were marked, and the transverse lengths of the immigrating cells from the initial wound were recorded [45].

### 2.8. Biological Properties of Nanoemulsion Wound Dressings Containing CA Leaf Extracts

The wound dressing was subjected to an evaluation of its biological activities (inhibition of adhesion, cytotoxicity, hemocompatibility, cell viability, cell proliferation, and cell migration assays, i.e., an *in vitro* scratch wound healing assay).

#### 2.8.1. *Ex Vivo* Antiadhesion Activity

This *ex vivo* experiment was performed as described in a previous study [46] with modifications. The susceptibility of bacteria to nanoemulsion wound dressings was determined by performing an antiadhesion assay. *S. aureus* (ATCC 25923) and *S. epidermidis* (TISTR 517) were cultured in TSB media. Then, they were incubated at 37°C for 4 h. Afterward, the inoculum was adjusted by 0.5 McFarland standards. The final concentration of inoculum was 5 × 10^5^ CFUs/ml. A 100 *µ*l drop aliquot of 10^5^ CFUs/ml (bacteria 10^4^ CFUs/pad) was used. The number of attached bacterial cells was evaluated at time points of 0 min, 1 h, 4 h, 12 h, and 24 h (5 time points). The nanoemulsion wound dressing (H, M, and L) was homogenized in a 1.5 ml Eppendorf tube containing 1 ml of a normal saline solution and serially diluted 10-fold in TSB. Then, 100 *µ*l of the bacterial suspension was spread on TSA and incubated at 37°C for 24 h. The test culture containing 1% DMSO was used as an untreated control. Finally, the bacteria were counted to determine the number of CFUs/ml at each time point.

#### 2.8.2. Cytotoxic Activity

The cytotoxicity of the CA extract was determined in a mouse fibroblast cell line (L929) using an SRB assay. The percentages of viable cells treated with the wound dressing containing three different concentrations of CA, namely, H (17.19 mg/ml), M (10.31 mg/ml), and *L* (3.44 mg/ml), are shown in Table 2. A blank wound dressing was used as a negative control. The cutoff percentage for cell viability indicating noncytotoxicity was greater than 80% [44].

#### 2.8.3. Hemocompatibility Assay

Hemocompatibility was verified using 2 methods. (1) CBC testing: a normal red blood cell (RBC) scatter Gram flag, as shown in Figure 3, was detected in the sample using the HA3 Hematology Analyzer (BioSystems, S.A.). The number of hemolyzed RBCs was quantitated from a normal RBC sample. RBC counts were adjusted to equal concentrations prior to an incubation with normal saline. If RBCs undergo hemolysis, normal RBCs would not be detected. In this test, DI water was used as a positive control. (2) Hemocompatibility test according to ISO 10993–4 [47]: this test was performed in an ISO 17025 laboratory (BioNEDD lab). This laboratory was approved by the Internal Review Board (IRB) at the Center of Ethical Reinforcement for Human Research of Mahidol University under ethical approval number 2018/007.0801. First, the total hemoglobin concentration in the blood sample was adjusted to 10 mg/ml by dilution with PBS after blood was collected from healthy human participants. Afterward, 1 ml of hemoglobin was added to 7 ml of samples from the three groups that were tested: normal saline (negative control), distilled water (positive control), and extract samples. The tubes containing the mixtures were incubated in a water bath for at least 3 back hours at 37°C and gently inverted every 30 minutes to mix. The mixture was then centrifuged for 15 minutes at 700–800 g. Subsequently, 1 ml of supernatant was mixed with 1 ml of Drabkin's reagent and the absorbance was measured at 540 nm with a UV-vis spectrometer. Equation (7) was used to compute the percentage of hemolysis as follows:

(7) $$\begin{array}{c} \text{hemolysis}\left(\text{\%}\right)=\frac{A^{S}-A^{B}}{\left(0.844\right)A^{T}-A^{B}}\times 100. \end{array}$$

#### 2.8.4. Cell Proliferation Assay

HDFs were used to determine the effect of the wound dressings on cell proliferation. First, HDFs were seeded in 96-well plates (1 × 10^4^ cells/well) and treated with different concentrations (H, M, and L) of the wound dressing. Second, cell proliferation was measured using the MTT assay. Normal media was used as a positive control, and a blank wound dressing was used as a negative control, as described previously [45].

#### 2.8.5. Cell Migration (*In Vitro* Scratch Wound Healing Assay)

HDFs were used to determine the effect of the wound dressing on cell migration. The cells were seeded in 24-well plates (5 × 10^4^ cells/well) using the protocol described above. The wound dressing contained different concentrations (H, M, and L). Then, the cells were photographed (Nikon Co. Ltd., Japan) on day 0, day 1, day 2, and day 3 and analyzed using ImageJ computing software. Normal media were used as a positive control, and a blank wound dressing was used as a negative control [45].

### 2.9. Statistical Analysis

For each sample, the findings are presented as the means ± S.E.M. of three determinations. Duncan's test was used to determine the statistical significance of differences in the data using SPSS statistics with one-way analysis of variance (ANOVA), and a *p value* less than 0.05 was declared significant.

## 3. Results and Discussion

### 3.1. Percent Yield of Extracts

DI water was used to extract CA by boiling. Each extract solution was evaporated to remove the DI water until it was dry, as shown by the constant weight. The resulting extract was frozen and freeze-dried for 24–48 h. The yield of the DI extract was 44.47% w/w. Therefore, a large amount of the leaves was extracted with water.

### 3.2. Calibration of CA Extract Concentrations

The spectrum for the CA extract is shown in Figure 1. The CA extract exhibited significant absorption signals at 286 and 288 nm. The peaks were located in the 270–290 nm region, which mainly represents total aromaticity involving *π* − *π∗* electron transitions, such as phenolic acids, benzoic acids, aniline derivatives, polyenes, and polycyclic aromatic hydrocarbons with two or more rings [48]. Wavelengths greater than 290 nm were excluded since no absorption signals were detected, and any absorbance values obtained at these wavelengths would have contributed a large amount of noise into the calibration matrix. Therefore, both wavelengths (286 and 288 nm) were used to determine the levels of CA extracts at pH 7.4 and pH 5.5, respectively, from a standard curve. The results of the standard curves obtained at pH 5.5 and 7.4 showed high accuracy between 0.05 and 0.5 mg/ml, with *R*^2^ values of 0.992 and 0.994, respectively. For the FTIR analysis, the round-shaped bands at 3,280 cm^−1^ (alcoholic O–H) [49], 2,920 cm^−1^ (alkanes C–H) [50], 1,593 cm^−1^ (cyclic alkene C=C) [51], 1,396 cm^−1^ (carboxylic acid O–H bending) [52], 1,253 cm^−1^ (aromatic ester C–O stretching) [53], 1,023 cm^−1^ (alkyl aryl ether C–O) [54], 887 cm^−1^ (alkyl aryl ether C–O bending) [55], and 665 cm^−1^ (alkene C=C) [56] indicate the presence of phenolic arenes and polycyclic aromatic hydrocarbons with two or more rings, consistent with the UV-vis spectrometry data. According to all the information mentioned above, most of the important substance of CA extract is probably physcion [57].

### 3.3. Preparation of CAN

The purpose of the FTIR spectroscopic investigation was to establish the chemical composition of CA extracts, the niosome surface, and the entrapment of CA extracts in niosomes. The FTIR spectra of the CA extracts are shown in Figure 4 (green line). Several stretching vibration bands associated with organic functional groups were clearly recognized in all of the spectra obtained. Round bands were observed at 3,280 cm^−1^, 2,920 cm^−1^, 1,593 cm^−1^, 1,396 cm^−1^, 1,253 cm^−1^, 1,023 cm^−1^, 887 cm^−1^, and 665 cm^−1^, which correspond to the vibrations of alcoholic O–H, alkane C–H, cyclic alkene C=C, carboxylic acid O–H bending, aromatic ester C–O stretching, alkyl aryl ether C–O, C–H bending, and alkene C=C [58]. The presence of phenolic arenes and polycyclic aromatic hydrocarbons with two or more rings was confirmed by the FTIR analysis, consistent with the UV‒vis spectrometry data. This result suggests that physcion is present [57].

Most critically, Figure 4 (red) shows the FTIR spectra of the freeze-dried niosome powder. In the niosome spectra, all peaks related to cholesterol and Span 60 were present. A few additional peaks were detected in the niosome spectra that were also visible in the cholesterol spectrum and Span 60 spectra. C–O stretching (1,060 cm^−1^), C–H bond stretching (2,952 cm^−1^), C–H bond bending (1,373 cm^−1^), and -OH stretching (a broad peak in the range of 3000–3700 cm^−1^) peaks were all visible in the cholesterol spectrum. C=O stretching (1,731 cm^−1^), -C-CO-O- (1180 cm^−1^), aliphatic CH stretching, asymmetric, and symmetric (2,914 cm^−1^ and 2,852 cm^−1^, respectively), and aliphatic -CH_2_- rocking (723 cm^−1^) peaks were observed in the Span 60 spectrum. The peaks observed for the CA extracts were detected in the CA-loaded noisome spectrum. The absence and decrease in the level of any peaks of CA extracts [59] when loaded in niosomes were confirmed by the FTIR spectra because the CA extracts were loaded in niosomes. Significant hydrogen bonding between formulation components is ascribed to a very broad peak that appeared in the region 3,000–3,700 cm^−1^, and the hydrogen bond is more likely to develop between CA extracts, cholesterol, and Span 60, according to previous studies [59].

### 3.4. Determination of the Size, PDI, and Vesicle Charge of CAN

The mean diameters, PDI, and charges of the niosomes prepared under the four conditions with various Span 60 weight ratios are shown in Figure 5. For all experimental settings evaluated, the results in Figure 5 show a clear correlation between the weight of Span 60 utilized and the resulting mean size of the niosomes (*p* < 0.05). The smallest mean size was observed for niosomes with a Span 60:cholesterol ratio of 3:1, while the largest average size was observed for niosomes with a Span 60:cholesterol ratio of 4:1. The 1:1 Span 60:cholesterol niosomes had mean diameters ranging from 226.2 to 236.6 nm, with an average of 231.4 nm, but the mean size of the 4:1 niosomes ranged from 479.9 to 493.9 nm, with an average of 486.9 nm. The average vesicle size was increased due to the increased weight of Span 60 due to the sorbitan esters of Span 60, which entrap soluble drugs in multilamellar vesicles. However, a larger amount of CA extract was loaded in niosomes containing a large amount of Span 60 than in niosomes containing a smaller amount of Span60. The EE and yields of Span 60:cholesterol niosomes prepared at a 4:1 ratio were low because the size was too large, resulting in precipitation. Furthermore, nonuniformity was discovered in the PDI of nanoparticles prepared at a 4:1 ratio, which was 0.489. A potential explanation for this result is that a PDI of approximately 0.3 is regarded as acceptable in drug delivery applications using lipid-based carriers, such as niosomes and nanoliposome formulations, and shows a homogeneous population of niosomal vesicles [60]. However, PDI values of 0.4 or higher are regarded as unsatisfactory and reflect a nonhomogeneous population. Notably, positively charged niosomes were reported to be toxic [61] and aggregate [62].

A negative charge causes electrostatic repulsion between particles, resulting in greater formulation stability [63]. However, the stability of particles strongly depended on Span 60 because highly negatively charged Span 60-containing niosomes bind many proteins, resulting in particle precipitation [64]. Therefore, a nonexcessive negative charge is suitable for niosome preparation. The results showed that the zeta potential of niosomes prepared using all ratios was negative, which might be explained by the adsorption of counter ions or the preferential adsorption of hydroxyl ions at the vesicle surface. The zeta potential values of niosomes with increasing Span 60 contents were higher than those with decreasing Span 60 contents because the high concentration of hydroxyl ions in Span 60 adsorbed on the surface of niosomes, resulting in a larger zeta potential [65].

As a result, the optimum Span 60:cholesterol ratio for the CAN was 1:1 because this ratio produces the maximum EE of 34.37% with an average size of 231.4 nm, a homogeneous solution with a good PDI of approximately 0.3, and less negatively charged niosomes.

### 3.5. Characterization of CANs

Niosomes were prepared with cholesterol and a nonionic surfactant to produce the amphiphilic structure of the membrane and provide stiffness and stability to the particles. CANs were effectively generated utilizing the thin film hydration process described in Section 2.4. CANs were analyzed for the following properties: yield, EE, and drug loading content. The optimal ratio of Span 60 to cholesterol was examined to produce the optimal niosomes, as shown in Table 3. Increasing the Span 60 ratio increased the drug loading content and EE. The 4:1 ratio resulted in the maximum drug loading and the largest size because the size was too large, causing precipitation. According to Table 3, a 1:1 proportion is adequate for the manufacture of CANs because it has the highest EE, high yields, and a nonnegative charge.

### 3.6. *In Vitro* Evaluation of CA Release from Niosomes

In the experiment, skin conditions were studied using the pH principle. The normal skin pH was determined to be 5.5, whereas the blood pH was 7.4. In Figure 6, CA release profiles from niosomes prepared with various proportions of Span 60 and cholesterol were evaluated at different pH values (pH 5.5 and pH 7.4). The release experiment was conducted in PBS (pH 5.5 and 7.4) with shaking at 37°C. As shown in Figure 6, pH 5.5, which is the pH of the skin surface, caused CA release. As a result, more than 80% of CA was released from 1:1 niosomes at pH 5.5 in 7 days, while only 60% was released at pH 7.4 in 7 days. Thus, CA would be released well on the skin (pH 5.5). However, it is less likely to be released in the blood (pH 7.4). Finally, it exhibits pH-dependent properties. When comparing the various niosome proportions, 1:1 niosomes exhibited faster CA release than the other proportions. When the Span 60 ratio was reduced, drug release increased. In contrast, as the Span 60 ratio increased, a slower release rate was observed. A potential explanation for this result is that Span 60 stabilizes niosomes and reduces niosome permeability to the encapsulated drug, reducing leakage. Thus, a 1:1 proportion was chosen for the synthesis of CA-loaded niosomes because CA release was the fastest and produced a sufficiently high level of inhibitory activity against human pathogenic bacteria. In the practical design for wound dressings, changing the dressing every 7 days is cost-effective compared to conventional dressings that must be replaced every 1–3 days [66].

### 3.7. Synthesis of A/P Hydrogels

The ideal quantity of calcium chloride was chosen based on the crosslinking percentage of CaCl_2_ and the contact time required for effective crosslinking of the films. The films that were crosslinked for 15 seconds with 0.5% w/v and 1% w/v calcium chloride solutions displayed good film homogeneity, were not brittle, and were smooth at the edges. Because the increased degree of crosslinking between the polymers led to a change in the physical appearance, the films crosslinked with 0.5% and 1% w/v crosslinking solutions for more than 15 seconds exhibited greater stiffness, brittleness, and less smooth edges with more wrinkles, as shown in Figure 2. Crosslinking times and concentrations greater than 15 seconds and 0.5% w/v were excluded to better characterize and analyze the durability of the films. The crosslinked films were prepared by incubating them with 1% w/v calcium chloride for 15 seconds during the entire study. Chemical crosslinking with the CaCl_2_ solution enabled soluble A/P hydrogel films to form hydrogel sheets that were insoluble. Intermolecular SA-to-PC connections are caused by Ca^2+^, which generates egg-box junctions necessary for the formation of PC and SA gels. Chemical bonds formed between the guluronate subunits of SA, galacturonate subunits of PC, and calcium ions are primarily responsible for the formation of the gel after crosslinking [67]. Because a plasticizing agent (in our case, glycerol) permits its flexibility even when it was dried at high temperatures, 7% glycerol was added to the crosslinked hydrogel film [68]. The approach of utilizing Ca^2+^ as a crosslinker for ionic polysaccharides has acquired universal acceptance and satisfaction. Therefore, the production of a polymer film crosslinked with Ca^2+^ improves its properties and is universally acceptable.

According to antibacterial activity and cytotoxicity, wound dressings were designed by considering drug release. Therefore, wound dressings were prepared that contained low (3.44 mg), medium (10.31 mg/ml), and high (17.19 mg/ml) doses of CANs.

### 3.8. Analysis of the Swelling Percentage

The effectiveness of the dressing in absorbing wound fluid and exudates is determined by the degree of swelling.  Figure 7 depicts the swelling behavior of A/P hydrogels as a function of time. Within the first 30 minutes, all samples showed a quick increase in the swelling degree, which continued slowly for up to 2 hours. Furthermore, as the alginate content in the hydrogels increased, the swelling degree decreased, which might be related to the structure of the alginate matrix that contains microscopic pores preventing water molecules from diffusing into the hydrogel structure. Previous studies [69, 70] reported similar behaviors for alginate-based hydrogels. The decrease in the swelling degree of hydrogel samples crosslinked with high calcium chloride concentrations indicates a strong hydrogel film, which is reported to be induced by Ca^2+^ leading to a model for zones of junctions popularly known as egg-box junctions necessary for the crosslinking of the A/P hydrogel. Furthermore, the presence of an ionizable COO-functional group can increase the volume between polymeric chains and the swelling capacity of the hydrogel through hydrostatic repulsion [71, 72]. The composition of A/P as 1/1 w/w crosslinked with 0.5% calcium chloride had the highest swelling degree of A/P hydrogels at 1,097%. In terms of water uptake, all swollen hydrogels had a maximum water content of 900–1,100%, showing that the A/P hydrogels would meet the requirements for an ideal wound dressing [73, 74] and protect wounds from fluid accumulation by absorbing exudates.

### 3.9. Biological Properties of CAN Wound Dressings

#### 3.9.1. Antimicrobial Activities

*(1) Agar Disc Diffusion Method*. The study was performed using an agar disc diffusion assay, and the extracts were used at concentrations of 4 and 8 mg/disc. The CA extracts exerted antibacterial effects on *S. aureus* and *S. epidermidis,* as shown in Table 4. The 4 and 8 mg/ml CA extracts showed strong inhibitory effects on *S. aureus* and *S. epidermidis,* with inhibition zones of 9.84 ± 0.14, 10.24 ± 0.34, 11.89 ± 0.93, and 14.08 ± 0.55 mm, respectively. The positive control oxacillin produced inhibition zones of 18.42 ± 1.33 and 26.85 ± 0.26 mm, respectively.

*(2) Broth Microdilution Method*. The antimicrobial activity of the sample extract was determined using the broth microdilution method to confirm the results from the agar disc diffusion method. The bacteria in this study were treated with different concentrations of each extract and standard drugs ranging from 16 to 0.25 mg/ml. The CA extract had an MIC of 0.5 mg/ml and MBC of 16 mg/ml against *S. aureus* and an MIC of 0.25 mg/ml and MBC of more than 16 mg/ml for *S. epidermidis.* The standard drugs still showed MIC and MBC values that were effective against the microbes (Table 5).

#### 3.9.2. Cytotoxic Activity

The SRB test relies on basic amino acids in the cells absorbing the negatively charged pink amino-xanthine dye SRB. The larger the number of cells is, the more dye is taken up, and when the cells are lysed after fixation, the liberated dye will have a stronger color and absorbance [44]. The results showed that cells treated with the CA extract at a concentration of 0.125 mg/ml had the highest viability at 95.32%, as shown in Table 6. Moreover, several concentrations of the CA extract, such as 0.125, 0.25, 0.5, and 1 mg/ml, resulted in greater than 80% cell viability. The results indicated that concentrations of the CA extract up to 1 mg/ml were not cytotoxic toward the L929 cell line.

For the nanoemulsion wound dressing, the results from the SRB assay found that the *L* nanoemulsion, which contained the lowest concentration, generated the highest percentage of cell viability at 89.56%. At the highest concentration, H showed the lowest percentage of cell viability at 87.29% (Table 6). Obviously, the percentage of cell viability was affected by the concentration of the crude CA extract, which was the active compound in the nanoemulsion wound dressing. However, all concentrations of the CA wound dressing that were mentioned above still showed a percentage of cell viability greater than 80%. Therefore, it was an acceptable value for the noncytotoxic effect on the L929 cell line [75].

#### 3.9.3. Cell Proliferation Assay

Cell proliferation was assessed using the MTT method. The CA extract exhibited a potent effect on proliferation (100.6–110.5%) at concentrations of 0.75, 1.56, 3.12, 6.25, and 12.5 *µ*g/ml, while the concentrations of 25, 50, and 100 *µ*g/ml exerted less of an effect on proliferation (75.9–88.8%). Furthermore, the highest percentage of migrating HDF cells treated with 3.12 *µ*g/ml CA extract was observed on day 3 (85.6%), as shown in Table 7 and Figure 8. The results showed that all of the concentrations displayed similar proproliferative activity to allantoin. Considering the high yield and good wound healing activity of CA, this extract was then selected further for the development of CA wound dressings. The analysis of the effect of the application of the CA wound dressing at concentrations ranging from 1.56 to 75% on proliferation revealed that the hydrogels at the concentrations were 3.12, 6.25%, and 12.5%. Cells grew much more quickly than the control, resulting in higher cell numbers than the control. HDF proliferation was significantly higher than that of the control group (*p* < 0.05). The proliferation of fibroblasts was equivalent to that of the positive control group treated with *Aloe vera* gel at a concentration of 12.5 *µ*g/ml. The proliferation of fibroblasts was 112.7% and 114.2%, respectively (Table 2). Thus, the proliferation assay revealed that all tested dosages of all formulations exhibited better activity in promoting the proliferation of HDFs than the gel base and *Aloe vera* gel.

#### 3.9.4. Cell Migration (*In Vitro* Scratch Wound Healing Assay)

The highest percent of HDF cell migration induced by the CA extract at concentrations of 1.56, 3.12, and 6.25 *µ*g/ml was observed on day 3 at 85.6%, followed by the CA extract at 6.25 *µ*g/ml (82.6%). The migration of the control group on day 3 was 51.4%. Moreover, the concentrations of 3.12 and 6.25 *µ*g/ml resulted in higher migration of HDF cells than the control and allantoin treatments. Cell migration induced by the CA extract and allantoin is shown in Table 7 and Figure 8.

The results obtained with the CA wound dressing showed that the wound dressing induced HDF migration (Figure 9; Table 7). Wound dressings at concentrations of *L*, M, and H induced the migration of HDFs. The highest cell migration occurred on day 3 after the administration of the test dose. The percentages of migrating HDFs treated with the three concentrations were 64.9%, 82.9%, and 82.4%, respectively. Moreover, all tested concentrations exerted a greater effect on the migration of HDFs than the gel base and *Aloe vera* gel. The results indicated that CA wound dressings might be useful for wound healing applications.

Statistically significant differences between control and various concentrations of sample were designated at *p* < 0.05. Dunnett's *t* tests treated one group as a control and compared all other groups with it (^*∗*^control; ^*∗∗*^allantoin; ^a^control; ^b^*Aloe vera* gel).

#### 3.9.5. Antiadhesion Activity

The effects of the wound dressing on the capacity of staphylococci to adhere to the epidermal tissue were studied using an *ex vivo* experiment, as shown in Figure 10. After 4 hours of treatment, the wound dressing at concentration H significantly reduced the number of adherent bacteria when compared to the control (*p* < 0.05). Moreover, the other concentrations (M and L) did not show the potential to inhibit bacterial adhesion. Although M was not able to reduce the adhesion of bacteria, it inhibited bacterial growth, as shown in Figure 10.

### 3.10. Hemocompatibility Assay

Since wound dressings were employed to cover the injury site, they directly contacted the blood. Therefore, they must be evaluated for hemolysis because of the prolonged contact throughout the wound healing phase. The hemolytic activity of wound dressings without the CA extract and wound dressings containing a low dose of 3.44 mg/ml, medium dose of 10.31 mg/ml, and high dose of 17.19 mg/ml CA extract are shown in Figure 3. The hemolytic activity was compared to that of the positive and negative controls. A nonhemolytic state is indicated by RBCs without hemolysis (negative control) of approximately 1.04 × 10^6^ cells/*µ*l. As a result, wound dressings containing the CA extract at 3.44 and 10.31 mg/ml had no effect on the hemolysis of human RBCs (1.06 × 10^6^ cells/*µ*l). Due to the release of a high dose of CA extract from the niosome, the wound dressing containing the high dose of the CA extract (17.19 mg/ml) had significant hemolytic activity, as shown in Figure 3(e). As a result, the hemolytic activity of wound dressings without the CA extract and wound dressings with low and medium doses of the CA extract were not significantly different (*p* < 0.05), but hemolytic activity between those wound dressings and wound dressings with high doses of CA extract were significantly different (*p* < 0.05). A greater number of RBCs were observed after treatment with wound dressings containing low and medium doses of the CA extract than after treatment with wound dressings containing high doses of the CA extract because wound dressings with low and medium doses of the CA extract prolonged and controlled the release of the CA extract safely and in the therapeutic range. The cumulative release of CA extract from wound dressings containing low and medium doses was 2.752 and 8.248 mg, which were calculated from 80% cumulative release in Figure 6(b), respectively, for 7 days. Furthermore, the hemolysis property was tested in accordance with ISO 10993. The wound dressing containing a medium dose of the CA extract was tasted. Wound dressings containing high concentrations of the CA extract had an effect on hemolysis, while the hemolytic grading of wound dressings with a medium dose of CA extract was 0.12 ± 0.05%. A nonhemolytic condition is indicated by a hemolytic index of less than two [76]. As a result, the wound dressing containing a medium dose of CA extract had no hemolytic activity and was recommended for development as a wound dressing.

## 4. Conclusions

In conclusion, a wound dressing prepared with CAN showed great potential when the Span 60:cholesterol ratio was 1:1. Then, 10.31 mg/ml (medium dosage) CA nanoparticles were used. A medium dosage is safe to use although it is less efficient than 17.19 mg/ml (high dose) at suppressing the growth of microorganisms. A medium dose did not affect RBC hemolysis, while a high dose resulted in hemolysis. Therefore, the medium dosage niosomes were then incorporated into wound dressings with A/P in a 1:1 ratio. Crosslinking was needed to strengthen the wound dressing. In the present study, crosslinking with 1% calcium chloride for 15 seconds maintained strength and form. This study will help produce wound dressings with appropriate physical and biological features. Animal (in vivo) and human safety (clinical phase 1 trial) and effectiveness investigations are needed (clinical phase 2 trial).

## Figures and Tables

**Figure 1:** UV absorption spectra of the CA extract at pH 5.5 (blue line) and pH 7.4 (red line).

**Figure 2:** Physical appearance of alginate/pectin hydrogel films crosslinked with CaCl_2_ concentrations of 0.5% and 1% (*Y* axis) for times ranging from 15 seconds to 120 seconds (*X* axis) compared to the control without crosslinking (a).

**Figure 3:** RBC histogram from the hemolytic activity test of (a) the negative control (normal saline) and (b) positive control (distilled water) and wound dressing containing (c) low, (d) medium, and (e) high doses of the water extract of CA leaves.

**Figure 4:** ATR-FTIR spectra of the niosome (red line), CA extract (green line), and CA leaf extract loaded in niosomes (blue line).

**Figure 5:** Characterization of nanoparticles. Particle size distribution of CA-loaded nanoparticles prepared at different ratios of Span 60 and cholesterol (1:1 (a), 2:1 (b), 3:1 (c), and 4:1 (d)) and zeta potential measurements of CA-loaded nanoparticles prepared at different ratios of Span 60 and cholesterol (1:1 (e), 2:1 (f), 3:1 (g), and 4:1 (h)) using a Zetasizer Nano ZS instrument (Malvern Instruments).

**Figure 6:** *In vitro* drug release profile of CA-loaded nanoparticles prepared at different ratios of Span 60 and Chol: 1:1 (red), 2:1 (blue), 3:1 (green), and 4:1 (orange) at pH 5.5 (square) and 1:1 (red), 2:1 (blue), 3:1 (green), and 4:1 (orange) at pH 7.4 (triangle) in terms of mg (a) and percent (b).

**Figure 7:** Swelling curves for wound dressings containing 1:1 A/P ratios with crosslinking using CaCl_2_ at 0.5% (red) and 1% (blue) in PBS, pH 7.4.

**Figure 8:** Effect of the water extract of CA leaves on HDF cell migration.

**Figure 9:** Effect of the wound dressing containing the water extract of CA leaves on HDF cell migration.

**Figure 10:** Kinetics for the inhibition of (a) *S. aureus* and (b) *S. epidermidis* attachment after treatment with wound dressings containing a high dose (red), medium dose (blue), and low dose (green) of the CA leaf extract compared to blank wound dressing (orange).

**Table 1:** Niosome formulations.

S:C ratio	CA (mg)	Span 60 (mg)	Cholesterol (mg)
1:1	10	5	5
2:1	10	6.6	3.4
3:1	10	7.5	2.5
4:1	10	8	2

**Table 2:** Effect of the water extract of CA leaves and CA wound dressing on HDF cell proliferation.

Samples	% cell proliferation after treatment with various concentrations (*µ*g/ml)								
	0	0.75	1.56	3.12	6.25	12.5	25	50	100
Control	100.0 ± 0.0								
CA extract		107.5 ± 1.1^*∗*^	110.5 ± 1.3^*∗*^	115.7 ± 2.9^*∗*^	108.8 ± 1.7^*∗*^	100.6 ± 1.9	88.8 ± 0.4	81.2 ± 1.5	75.9 ± 1.3
Allantoin		108.1 ± 1.5^*∗*^	113.5 ± 2.8^*∗*^	115.4 ± 1.8^*∗*^	111.5 ± 2.3^*∗*^	106.8 ± 2.5	90.7 ± 1.5	85.3 ± 2.4	74.0 ± 2.7

	% cell proliferation after treatment with various concentrations (% of the wound dressing)								
	0	1.56	3.12	6.25	12.5	25	50	75	

Control	100.0 ± 0.0								
CA wound dressing		97.4 ± 1.5	105.5 ± 1.7	112.7 ± .4^*∗*^	102.3 ± 2.8	91.3 ± 1.6	81.7 ± 1.5	72.7 ± 5.6	

		% cell proliferation at various concentration (*µ*g/ml)							
	0	1.56	3.12	6.25	12.5	25	50	100	

*Aloe vera* gel		93.8 ± 3.7	98.6 ± 0.9	103.4 ± 2.1	114.2 ± 1.2^*∗*^	95.8 ± 0.7	96.4 ± 0.6	90.0 ± 2.5	

Each value represents the mean ± S.E.M. of three determinations. ^*∗*^Statistically significant differences between the control and various concentrations of sample at the 0.05 level. Dunnett's *t* tests treated one group as a control and compared all other groups with it.

**Table 3:** Drug loading capability of CA leaf extract loaded in niosomes prepared with four different ratios of Span 60 to cholesterol.

S:C ratio	Drug loading (%)	EE (%)	Yield (%)
1:1	8.56 ± 0.32	34.37 ± 3.34	57.62 ± 7.59
2:1	7.42 ± 0.55	31.83 ± 1.43	61.43 ± 2.02
3:1	6.90 ± 0.50	16.90 ± 4.40	34.76 ± 8.19
4:1	12.30 ± 1.05	13.87 ± 1.20	16.19 ± 1.78

**Table 4:** Antibacterial activity of the CA leaf extract assessed using the agar disc diffusion method.

Bacteria	Efficacy of bacteria inhibition							
	4 mg/ml		8 mg/ml		Positive control*∗*		Negative control	
	Clear zone (mean ± SD) (mm)	Susceptibility test	Clear zone (mean ± SD) (mm)	Susceptibility test	Clear zone (mean ± SD) (mm)	Susceptibility test	Clear zone (mean ± SD) (mm)	Susceptibility test
*S. aureus*	9.84 ± 0.14	I	11.89 ± 0.93	S	18.42 ± 1.33	S	—	—
*S. epidermidis*	10.24 ± 0.34	I	14.08 ± 0.55	S	26.85 ± 0.26	S	—	—

Standard drug: oxacillin for *S. aureus* and *S. epidermidis*.

**Table 5:** Antibacterial activity of the CA leaf extract as assessed using the broth microdilution method.

Bacteria	Efficacy of bacterial inhibition					
	CA extract		^*∗*^Positive control		Negative control	
	MIC	MBC	MIC	MBC	MIC	MBC
*S. aureus*	4 mg/ml	16 mg/ml	0.5 *µ*g/ml	1 *µ*g/ml	—	—
*S. epidermidis*	1 mg/ml	>16 mg/ml	0.25 *µ*g/ml	0.25 *µ*g/ml	—	—

^*∗*^Standard drug: oxacillin for *S. aureus* and *S. epidermidis*.

**Table 6:** Effectiveness of the CA leaf extract and CA wound dressing on L929 cell viability.

Sample	Concentration	Percentage of cell viability ^*∗*^(%)
CA extract	2 mg/ml	65.47 ± 1.42
	1 mg/ml	81.32 ± 2.16
	0.5 mg/ml	89.88 ± 1.98
	0.25 mg/ml	94.76 ± 2.75
	0.125 mg/ml	95.32 ± 0.57

Control of CA extract	—	104.28 ± 2.37

CA wound dressing	H *µ*g/ml	87.29 ± 1.67
	M *µ*g/ml	87.55 ± 1.95
	L *µ*g/ml	89.56 ± 2.03

Control CA wound dressing	—	102.02 ± 3.07

Negative control CA wound dressing ^*∗∗*^	—	101.97 ± 2.44

^*∗*^Results are presented as the means ± SD of three independent determinations (*N* *=* *3*); ^*∗∗*^negative control (blank wound dressing).

**Table 7:** Effect of the water extract of CA leaves and CA wound dressing on HDF cell migration.

Samples	Concentration (*µ*g/ml)	Length between the scratch (*µ*m)				% migration rate of cells			
		Day 0	Day 1	Day 2	Day 3	Day 1		Day 2	Day 3
Control	—	1131.5 ± 52.7	921.4 ± 26.0	734.0 ± 25.3	493.8 ± 44.0	18.4 ± 1.8		35.0 ± 0.9	51.4 ± 2.8
CA extract	1.56	995.4 ± 16.8	793.2 ± 23.3	510.2 ± 71.6	251.0 ± 16.7	20.4 ± 1.0		48.6 ± 7.9	73.6 ± 1.6^*∗*^
CA extract	3.12	1030 ± 48.7	716.5 ± 42.3	483.4 ± 50.7	147.9 ± 2.4	30.4 ± 3.5^*∗*^		52.6 ± 5.1	85.6 ± 0.8^*∗*^
CA extract	6.25	995.3 ± 21.0	752.7 ± 14.3	501.9 ± 54.1	166.5 ± 17.8	21.1 ± 2.6		46.1 ± 5.9	82.6 ± 1.9^*∗*^,^*∗∗*^
Allantoin	3.13	1084.5 ± 77.3	813.9 ± 28.9	589.0 ± 61.6	342.3 ± 22.0	24.6 ± 2.8		45.7 ± 3.6	68.4 ± 0.5^*∗*^,^*∗∗*^
	% of wound dressing	Length between the scratch (*µ*m)				% migration rate of cells			
Control	—	872.7 ± 24.1	793.1 ± 39.7	591.2 ± 47.8	373.2 ± 2.2	8.9 ± 5.8	32.4 ± 4.0		54.3 ± 2.3
CA wound dressing	3.12	1028.3 ± 29.9	861.7 ± 25.9	653.0 ± 25.4	396.5 ± 13.1	16.2 ± 1.2	36.5 ± 1.6		64.9 ± 2.6a
CA wound dressing	6.25	979.2 ± 17.0	832.6 ± 17.6	571.0 ± 20.6	167.1 ± 4.8	14.9 ± 3.0	40.9 ± 0.7a		82.9 ± 0.4a, b
CA wound dressing	12.5	999.0 ± 19.8	887.3 ± 50.2	593.8 ± 22.9	175.7 ± 10.0	11.3 ± 3.6	38.3 ± 2.2		82.4 ± 1.3a, b
*Aloe vera* gel (*µ*g/ml)	12.5	1028.1 ± 22.6	799.7 ± 11.5	556.3 ± 24.5	227.2 ± 12.2	22.1 ± 0.7a	45.9 ± 1.8a		73.1 ± 0.9 b

Each value represents the mean ± S.E.M. of three determinations.

## Data Availability

The data used to support the findings of this study are included within the article.
